RETRACTED

# Deep-Learning-Guided Student Intelligent Classroom Management System

**DOI:** 10.1155/2022/1961631

**Published:** 2022-08-26

**Authors:** Xiaobing Niu

**Affiliations:** Zhengzhou Preschool Education College, Zhengzhou 450000, China

## Abstract

Aiming at the limitations of old-fashioned instructing knowledge and the insufficiency of existing dynamically managed classrooms, a deep-learning-guided Unity3D-based intelligent classroom management system and the corresponding instrument support were proposed. We first build a virtual scene and import Unity3D motors, in order to improve practical fake action proofs through C# script and prefix system. Subsequently, we attempt to solve the permission arrangement proposition in multiperson entity scenes, and accordingly, we complete the cognitive assistance module using authorization strategy. Our system can provide different students with tailored permissions, foresee text, video, and some flexible functions. Our system can be divided into multiple Spring Cloud frameworks. We further leverage the Redis to optimize the system architecture. The system can be conveniently applied in chemistry instructing with clear virtual auditions under the government direct supervision. It can effectively address authority issues in real scenarios while enhancing the learning efficiency and increasing accessibility. A set of intelligent classroom behavior system based on deep learning that supported by cunning learning methods are proposed accordingly. It can complete the classroom perception ministry. It can optimally conduct status monitoring as well as classroom assignment and discussion services through deep learning vision techniques such as face perception and facial expression analysis. Extensive experimental results have shown the competitive performance of our method.

## 1. Introduction

Intelligent classroom instructing is the key platform for the cultivation of professional talents in various colleges and universities. In practice, all colleges and universities pay great attention to it [1–5]. The current manual management operation typically utilizes various means such as attendance and classroom performance evaluation. These techniques have many shortcomings such as low efficiency and insufficient evaluation. Many colleges and universities have attempted to apply various software to encourage students to attend the classroom. However, such a mechanism cannot successfully solve the serious problems of low classroom efficiency such as students' unwillingness to participate the classroom and their disinterest in the learning content. For example, instructors at Chongqing University use fingerprint attendance [1], and students utilize fingerprint punch-in machines to check in and check out. Meanwhile, instructors from the Zhuhai College of Jilin University have developed a set of Bluetooth-based attendance systems, which are matched with students' Bluetooth devices before class. In addition, there are many ways to scan QR code to sign in, send Weibo to sign in, check in and check in. We in this paper propose an intelligent classroom management framework, which realizes the function of classroom check-in through deep-learning-based face detection. We further evaluate students' relevant learning emotional status by recognizing facial expressions. The results of system evaluation and related data analysis have demonstrated that the system is useful for instructors to evaluate students' individual learning performance in a timely and objective manner. Simultaneously, it is convenient for instructors to improve their instructing experiences based on the course targets and learning atmosphere.

RETRACTED

The experimental results of the “Survey Report on Online Teaching of College Teachers During the Epidemic Period” and the “Survey Report on Online Learning of College Students” are illustrated in the following [6–13]. This is conducted during the Epidemic [3] trial by the Teacher Development Center as well as the protect of this researches. The problems existing in the implementation of online road at colleges and universities can be summarized as syn: “Students are weak in autonomous learning,” “Part of the teaching content is not suitable for online teaching,” “‘Live broadcast + online interaction' is the main mode of online teaching,” “Insufficient student participation,” “teaching evaluation methods and methods are not becoming for online teaching,” and so on. To well explain the key problems existing in the implementation of online career in colleges and universities during the epidemic period, and on the base of multidisciplinary speculation, we in this paper intend the design concepts that are motivated by the implementation of online method in colleges and universities. Carl Rogers, an American psychologist, put prompt “learner-centred” conception, which center on empowering learners to study independently. This theory focuses on the positive interaction between instructors and students' emotions and cognition and the development of a good learning situation and atmosphere. The model is designed based on the concept of “learner-centered.” It can not only follow the Carl Rogers' proposition but also further highlight what it is centered on cultivating students' learning capacity. Learning capability is a combination of self-transformation, innovation, and development of learners' learning motivation, learning perseverance, and learning ability. The data calculated during the epidemic period have optimally shown the autonomous learning ability of college students in our country, that is, the learning capacity of college students, is relatively weak. Therefore, the model design of online courses should be learner-centered, and the learning process should be carried out around cultivating learners' autonomous learning ability. Our method highlights the problem of current college students' learning as well as the problem of power lacking.

RETRACTED

In this work, we implement a deep learning framework of college online courses management. The model focuses on optimizing learner and is guided by deep learning. The entire framework includes the deep learning pretraining stage, the deep knowledge refinement stage, and its evaluation stage. Model refinement reflects the learner-centered position of curriculum design and the model-oriented distribution of curriculum resources. It includes the in-depth learning as the benchmark for the level of curriculum teaching, as well as the multiline interaction as the connection for the organization of curriculum activities. It also provides multiple practical approaches for curriculum practice. Self-learning is the driving force, the design of the course is supported by the learning techniques, and the expansion of the course spatially and temporally is based on ubiquitous learning. Meanwhile, the development of academic evaluation is based on the panoramic perspective. Afterward, the model is applied to the particular course implementation through active research, wherein comprehensive experimental results have shown that this model can effectively avoid the typical problems in online teaching. Meanwhile, it can also effectively promote students' in-depth learning. This can achieve the best learning performance.

## 2. Related Work

“Live broadcast + online interaction” is the main mode of online instruction in colleges and universities during the epidemic [7–16]. According to Bloom's plan of the goal dimension in the cognitive domain, the cognitive goal of “live broadcast + online interaction” is still in the shallow learning stage of “knowing and understanding.” Comparatively, the deep learning is built upon cultivating learners' higher-order thinking ability of “application, analysis, synthesis and evaluation.” The instructing method of the school has not been clearly implemented in the online teaching of colleges and universities during the epidemic. Eric Jensen and LeAnn Nickels-en, the two well-known American scholars and teachers' vocational trainers, proposed the route of Deep-per Learning Cycle (DELC) from the perspective of teachers' instructing, the DELC route. The above operations consist of seven steps: designing standards and curriculum, preassessment, creating a positive learning culture, activating prior knowledge, acquiring new knowledge, processing knowledge in depth, and evaluating students' learning according to the DELC route and online colleges during the operation. Instruction is generally in the reality of shallow learning, and the model design of online courses takes deep learning during the implementation stage.

RETRACTED

Michael G. Moore's Theory of Transactional Distance (Theory of Transactional Distance) believes that [10–18] interactional distance refers to the distance at which physical distance leads to the potential psychological or communication misunderstandings. Interaction distance is directly affected by three types of variables: dialogue, structure, and autonomous learning. During the epidemic, the lack of student participation in online courses in colleges and universities has demonstrated that due to insufficient instructor-student dialogue. It lacks the flexible course design structure and weak learner autonomy. The interaction distance has affected students significantly. The focus of interactive learning is to promote the interaction between teachers and students, students, and groups, with the support of information technology and the interaction as the core feature. Through multiline interaction, learners interact with various elements in the learning environment. We can build a learning community and make learners feel the results of interaction such as thoughts and emotions. M • Carolyn Clark, a well-known educational scholar who first proposed the concept of embodied learning theory, believed that embodied learning is not a kind of conscious learning. He refers to the physical stimulation of daily life or work through feeling rather than changing the psychological and emotional level. This in turn responds through the body [7]. Embodied learning emphasizes learning through body perception and experience in the process of interaction between the body and the environment. We leverage embodied learning to carry out practical activities of online course teaching, which is beneficial to learners to deeply understand the knowledge they have learned.

Zhang et al., Bernard et al, and Chen et al. cited the construction industry's “bracket” [14–16] and then defined it in education as providing assistance to students according to their requirements and withdrawing help as they grow. The area where students' actual development level and potential development level overlap is called “zone of proximal development.” This is the region where students penury “verify” to complete the undertaking. The design of the online succession model in colleges and universities should take into narration all the possible difficulties that learners will encounter in the process of online self-governing learning and provide essential materials suitably to help learners acquire knowledge. U-Learning, as the name suggests, refers to intercommunication at all times and omnipresent lore, which is a journey for everyone to obtain any message they necessity, anywhere, at any tense. The target is to leverage information technology to provide students with a 4A (anyone, anytime, anywhere, and any device) learning platform that can be utilized anywhere and anytime to conduct learning activities with the tools at hand. Unlimited time and unlimited opening of learning resources in our context can reflect the characteristics of ubiquitous learning such as learning anytime, anywhere, unrestricted access to resources, socialization and personalization of cognitive networks, and the autonomous learning.

RETRACTED

## 3. Our Proposed Method

During the deep scholarship preparation stage, we conducted the enlightenment deep prominence stage and wise letter evaluation station. The projection system is an encircling system above the spiral, and the feedback from the previous program is carried out for the optimization of the next execution. The first bells and whistles are the preparatory stages of deep literature. Instructors are poor in front of the established exam learners and have also developed exam syllabuses. Prestandard learners are based on the support of systems and resources, and instructors conduct research on learner characteristics, beginners' situational characteristics, learner preferences, learner behavior characteristics, and exploration and utilization and other scholar means. Herein, we formulate a scholar model. The stigma of the preset curriculum is that instructors build knowledge models and doctrinal strategy dummies based on the cultivation of systems and resources.

The main links of learning mode interception are as follows: formulating curriculum goals and cherishing higher-order thinking and identifying challenging learning topics. We propose some ingenious questions that trigger cognitive struggles and configure multidimensional academic integration resources that connect contexts. The tactical mode of educating people is a synthesis of the instructing methods that conform to the characteristics of subordinates, the educating methods that conform to the teaching laws, and the educating methods that conform to the sects of scholars. Through the integration of the beginner mode, the acquaintance mode, and the instructing strategy mode, a variety of curriculum methods suitable for learners are constructed. The second stage is the in-depth scholarship process is conducted accordingly. That is, with the support of letter brackets and a complete knowledge chain, deep science becomes clear, and the learner's higher-order thinking efficiency is improved accordingly. The incomplete processing of acquaintances follows the progressive operations of stimulating old knowledge, making new friends, and connecting novel and original knowledge, knowledge construction and transformation, and cognitive creation.

RETRACTED

The technical process of the system is shown as follows. The client has been improved with Unity3D. The Shader for sofa rendering and control dummy material is provided, by leveraging the GUI as the interactive interface. The core secant line of the actual classroom is completed in business response, including user registration and login, the potential experimental server is developed with IDEA. And the client transmits it to the salver through the HTTP interface and applies the permission policy. MySQL is rich in persistent data like basic student ads, and Redis is rich in hot data as a hoard. When building the model, it is necessary to guarantee the determinism of the pattern. We should simultaneously ensure that the composition calculation of the vertices and the total number of virtual triangle parts are not too high, in order to avoid a lot of memory overhead at runtime. If the system has money, it will affect the inefficiency of the system. We have to make high-quality products such as test tools, fashion, and sophistication not influenced by occasions, classroom walls, etc. When the model is larger, reduce the fineness of the plane. After the model is generated, textures are incorporated to its material structure properties to calculate the simulated optical results. In addition, confirming a 1 : 1 ratio of potential scenery to real classrooms is essential to improve students' ability to unitize the system.

After the system is running, the strength glasses that can be used to log in are introduced in this section. This view is achieved through GUI, that is, a graphical user interface. Users control menus and icons on the screen through input devices such as a mouse to complete a series of interactions. The active GUI includes properties such as sections, buttons, and input boxes. After supplementing the interface, we combine the C# script components so that the UI can be leveraged for input. After the user clicks the login button, the system will judge whether it matches the existing data in the database according to the user input information and password text box. If the input usage information corresponds, the SceneManager.LoadScene() system API is called regularly through the Invoke() function to trigger the loading of the virtual classroom scene, and an original success message is quickly generated, otherwise, the usage input is cleared and a red error messenger is output.

RETRACTED

Face detection is mainly based on the MTCNN algorithm rules [3], involving neural networks and convolutional neural networks. The algorithm uses three subnetworks, namely, P-NET, R-NET and O-NET. P-NET: the network form mainly has the executing window of the epitaxial region and the regression vector of the boundary spar. And the bounding boxes will be regressed. Thereafter, the qualified small windows are graded, and subsequently, highly overlapping candidate boxes are merged through the nonmaximum barrier (NMS function). R-Net: the cobweb configuration will remove those unreliable provinces via bounding box regression and NMS. Due to the difference between the plexus structure and the P-Net network structure, incorporating a completely additional layer will achieve the correction effect of hiding fakes. O-Net: this layer has one more volute lift than R-Net lift, and the calculated results will be highly refined.

This R-Net technique has more superintendence on the facial extent and also production five instant. The processing of the latter coping is more delicate than the prosecute of the fore sill. Meanwhile, the production appearance information will be more accurate, and in the end, more instructive visual features will be origin. This scheme also uses the opencv algorithm government, basic affair trading operations for similarity reading, list, and storage. We call the cv2 in OpenCV. read(), cv2. imshow(), and cv2. print() is fulfill apar. The edifice sketch of the confederated algorithm MTCNN of this system is elaborated in the following. The cross-entropy injury is calculated as

(1) $$\begin{array}{c} L=-\left[y\log\left(p\right)+\left(1-y\right)\left\{1-\log\left(p\right)\right\}\right], \end{array}$$

The plexus-guided probability in the *p* example indicates that the image perceived currently is a face, and *y* denotes the test copy shameless exact label. Herein, *y* ∈ {0, 1}.

The aforementioned system has a big proposition: face alignment technology. In actual recourse scenarios, the grasping surfaces may be competitive, inclined, sideways, etc. In order to make the detection marks larger, the thickness will be corrected by a second-hand alignment technique. Face alignment is modeled shamelessly in the first place, which can be divided into global presence and local arrival modeling methods, such as the appearance model. Before generating shape, feature fashion [4], the above techniques are more typical alarm presence models. We consider how to extract the face appearance information modeling and upcoming provincial information modeling, including similarity models, projection models, and contour rope standards. We purpose the combining mtcnn algorithm to implement the existence alignment technique. We plan to obtain the tangent formed by the two views and the wheel—shape the appearance according to this angle. We try to get the rotated representation to appreciate the height of the face that must be cropped and further prevent the width ratio from determining the crop confidence width to obtain specific coordinates to perform face alignment.

RETRACTED

The MXNET library supports squeeze analysis of secant lines and can decompose the face declarations by leveraging multiple convolutional neural networks [5]. Among the nicknames for facial expression recognition, CK++ and MMI databases appeared in the recent ALICE, and databases such as Affectnet, AFEW-VA, and SFEW appeared in the low years. The face portraits in these databases have no requirements on the environment, including model sets of different locations and different denominations. In the facial shape extraction station, the existence feature point discovery is conducted in the first place, followed by the appearance alignment technique, and finally, the corresponding features are extracted. The appearance analysis refers to the front face is leveraged to eliminate a series of surrogates such as headgear pose and facial personalization [6] to obtain renormalized facial feature assignments. This results in shameless facial feature vectors as well as the expression confirmation.

## 4. Experimental Results and Analysis

This investigation adopts the method of action and deliberation and takes the online course “Basics of Elementary Education” as the practical treatment.

The deep learning university online course implementation mode carries out course planning and implementation, continuously improves learning methods, and promotes learners' autonomous learning and cooperative learning, so as to obtain profound knowledge. The test target of this activity is H University 2018 undergraduates of Chinese Language and Literature and Chinese to Speakers of Other Languages, a total of 87 adults. The action research period is the second semester of the 2019-2020 Plato academic year. The results of program implementation were analyzed through a combination of literature process performance and assessment questionnaires.

Learning process grades: the chief data self-possessed in this agency ponder learning process behavior are 12 correct assignments, of which the first 7 are extravertive debate, and the last 5 are objective interrogation. From the quantitative analysis point of scene, the realization of homework everywhere is useful, the average score of everywhere is around 88.5, and the mean worthy standard is around 59%, evince that most of the students have ended the goal of the chief's learning extend and capability training, and the scholarship performance is admirable. Nuts and bolts are shown in Table 1.

RETRACTED

Questionnaire view results: the five-level Likert ladder was chiefly employment in this behavioral assessment questionnaire, describe from “firmly disagree” to “vehemently harmonize.” This thinking uses SPSS22.0 software to decay the firm and intenseness of the evaluation questionnaire (expel unprejudiced dispute), where *a* = 0.914, the Cronbach's Alpha coöperating of each scope subscale is between 0.894 and 0.960, which relate the proud reliability of the questionnaire. The KM0 value was 0.895, and the questionnaire was found to have exalted robustness. The questionnaires were analyzed by commonality analysis, and the results are shown in Table 1. From the scenario of point 1, 72.29% of the “firm transaction” and 24.1% of the “correspondence” mode and a Go score of 4.69 imply that this approach works well for “learner-centric” dummy positioning. From the moment of the 2nd scenario, 68.67% “strongly agree” and 25.3% “agree” relish and 4.63 Norma charges, it is found that this method has a better allocation effect of course resources with scholar characteristics. From the details of topic selection, 73.49% of the “very fit” samples and 19.28% of the “harmonious” samples have a Go score of 4.66, indicating that this course adopts a generalist teaching model, which is more efficient in the allocation of course funds. Starting with the cliché 4 opinion, 68.67% “strongly agree” and 26.51% “agree” attempts and a running total score of 4.63, specifically stating that the implementation of this course performs better with the evenness and effect of convinced. From item 5, 71.08% “strongly agree” and 22.89% “agree”, with an average charge of 4.65. This sample demonstrates the intent and implementation of this legacy of knowledge scaffolding and supports students with competent letters. Judging from the remaining 6, 59.04% “strongly agree” and 26.51% “agree” samples and a Norma score of 4.45, it is found that the enflesh learning link proposed in this progress is more effective than in-body learning and can be achieved pure literature. Influences. From the scene of detail 7, 75.9% of the “strongly agree” and 20.48% of the “agree” test paper and standard score 4.72, solves this road, we solve this road and make up for the deficiencies of online erudition caused by separation of teachers and students, divorce between students and scenes through the flexible design of multidirectional interaction. From the 8-detailed inspection committee, a 75.9% “strongly agree” and 18.07% “agree” sample and an average record of 4.7 indicate that this course has created an admirable literary atmosphere by assembling cooperation letters, etc. From the details of item 9, 84.34% of the “extraordinary contracts” and 14.46% of the “commitment” samples, as well as the Norma Bill of 4.93, all show that the implementation mark of this course has certain advantages and is deeply loved by users. The average “very suitable” ratio of 9 questions is 72.15%, and everywhere is 4.67, indicating that the course correctly implements the concept of model mean, and the implementation effect is excellent.

RETRACTED

Judging from the achievements of the knowledge process and the results of the questionnaire survey, the implementation mode of online courses in colleges and universities based on complex learning can play a greater role.

The curriculum funding arrangement supported by the learner model, teaching strategy, and other forms is full of vitality, which can cherish the learners' higher thinking agility; the mode activity system can realize multitone interaction and harmonious learning; give learners equal support. Its implementation operations deceive the deep lore unit. It can be seen that this example can realize the design concept and achieve excellent results, which can explain the common problems in the implementation of online routing in colleges and universities, and has undoubted significance for recourse and promotion. Due to the limitations of repeated endings, sketch arrangement, and design methods, this research is still in the investigation stage, and it is necessary to continuously optimize and deepen in future teaching strategies.

Due to the incomplete interpretation of virtual reality in teaching applications and the failure of interactive permission control, this system proposes a dynamic permission control strategy based on RBAC support in a virtual environment. Commanders include users, roles, models, permissions, and events. 5 larger units, of which roles, fashion, and permissions are divided into fine-grained departments. A character one, a party in a vibrant landscape, holds three cues: a character identifier, a party name, and a party example. Different straightforward role types are different, such as bookman and index roles; there are also different party constitutions at the same level, such as common mining and monitoring roles. Model 1, the model in the virtual presentation, contains 4 sets of information: example identifiers, virtual permissions, and practice boundaries. Permissions unit refers to the permissions of roles and forks in the virtual exhibition, including 4 individual information: permission identification, direct permission, favorite content, and tolerance constraints. Permission satisfaction is divided into role management and model direction. Permission constraints include quantity constraints and time constraints, which are relatively limited. The maximum number of filled roles and the maximum disposition time of the reason prevents the “master.” The occurrence supervision mechanism is used to monitor all events in the virtual scene and process them according to event types and processing principles. In order to explain that the virtual multiplayer exhibition solves the handicap problem of actual design, the business ethics guidelines are put forward: (1) the principle of weighing priority, when the actual person does not practice the model interaction request, the node with the earlier opportunity for the party will have the correct model interaction. (2) The principle of authorization priority. For model interaction, when a role with other permissions starts a model interaction request at the same time node (opportunity interval is less than 1 ms), the party with higher authority will have priority in the model interaction vertical. (3) Scope assignment axioms, accustomed to refuting roles with the same authority at the same rhythm, nodes have not tried modulo interaction requests and caused the system to fail, and use random match numbers to solve the problem. In order to solve the moral bifurcation and attribution proposition without experimental arrangement in the multianthropomorphic environment, the class progress axiom is proposed: the student's role achievement and grade progress are combined to calculate the advantage antecedent value *T*, and the actual operation of the small *T* must first interact directly with the instance. Scholar's privilege priority value *s* *Ts* = (*ps*/*p*)*wp* + (*gs*/*g*)*wg*, *ps* is the positive utility of student role *s*. All student roles, *gs* is the course change of student party *s*, and *g* is all student roles. The scale course brand, *wp* is the weight of the class circuit on *T*, *wg* is the load of the grade on the value of *T*, and the system regulates the *T* respecting all potential roles by starting with this, arranging them into a queue in skewed order, and then dequeuing to grant permissions. The specific implementation of the above axioms relies on the update feature of the Unity3D batch file Update() method, each design, wearing this feature, it detects the event monitoring mechanism, continuously monitors the interaction request, and passes the HTTP interface including prayer time.

RETRACTED

## 5. Conclusions

On the basis of deep learning convolutional neural network, this project has done a great job in improving the efficiency of the classroom, reducing the teacher's task, supervising the students to study independently and self-discipline, and making it convenient for the instructor to understand the classroom situation, record the classroom, and analyze it at any time. The emotional state of the students facilitates the realization of related functions such as communication. The actual application has shown that the system runs stably and reliably and has high practical value.

## Figures and Tables

**Table 1:** Homework average scores and the excellent proportion.

	H1	H2	H3	H4	H5	H6	H7
Ave	0.763	0.804	0.863	0.783	0.882	0.789	0.881
Exl	0.641	0.621	0.573	0.643	0.583	0.582	0.627

## Data Availability

The relevant data can be obtained according to the request of the readers.
